The article "miR-100-5p Is a Novel Biomarker That Suppresses the Proliferation, Migration, and Invasion in Skin Cutaneous Melanoma" was retracted in 2023. Reasons: signs of a paper mill; suspected computer-generated content; unreliable results or conclusions; lack of ethics approval or compliance.

# miR-100-5p Is a Novel Biomarker That Suppresses the Proliferation, Migration, and Invasion in Skin Cutaneous Melanoma

**DOI:** 10.1155/2022/3585540

**Published:** 2022-09-20

**Authors:** Xiao Zhang, Yuqi Deng, Xiao Liang, Yamin Rao, Haiyan Zheng, Fei Liu, Xusong Luo, Jun Yang, Jun Chen, Di Sun

**Affiliations:** ^1^Department of Plastic and Reconstructive Surgery, Shanghai Ninth People's Hospital, Shanghai Jiao Tong University School of Medicine, Shanghai 200011, China; ^2^Department of Pathology, Shanghai Ninth People's Hospital, Affiliated to Shanghai Jiaotong University School of Medicine, Shanghai 200011, China; ^3^Department of Dermatology, Shanghai Ninth People's Hospital, Affiliated to Shanghai Jiaotong University School of Medicine, Shanghai 200011, China

## Abstract

**Objective:**

To better understand the role and underlying mechanisms of SKCM, we conducted bioinformatics analysis and in vivo experiments.

**Results:**

We found its role as a tumor suppressor gene in SKCM and its effect on prognosis. In addition, this study found that miR-100-5p had a bidirectional effect on SKCM microenvironment. After exploring the relationship between the two, it was found that tumors with intermediate miR-100-5p expression had the highest level of immune cell infiltration. In addition, the value of miR-100-5p was assessed by survival analysis, univariate Cox regression analysis, and nomogram prognostic prediction. Finally, we constructed a regulatory network to illustrate the regulatory relationship of miR-100-5p.

**Conclusions:**

In conclusion, the antitumor effect of miR-100-5p is revealed, and the present study is followed by a discussion of its molecular regulatory network, followed by novel insights into SKCM therapy.

## 1. Introduction

As one of the most ordinary deadly forms of skin malignancies in humans, cutaneous melanoma (SKCM) accounts for approximately 5% of all skin tumors [1]. DNA damage in melanocytes is the basic cause of malignant melanoma. On the basis of genetic background, long-term ultraviolet irradiation, repeated friction, and trauma stimulation lead to DNA fragmentation, translocation, mutation, or abnormal methylation of melanocytes. Melanocytes show uncontrolled proliferation and abnormal differentiation and finally develop into malignant tumor cells. Meanwhile, it is responsible for more than 80% of all skin cancer-related death, and the mortality rate rises annually [2]. Surgical resection is the most effective therapeutic option for the early stage of SKCM. However, its invasive and aggressive properties lead to a poor prognosis. As a result, investigating molecular mechanisms was crucial, which might help explain the tumorigenesis and development of SKCM. In order to better explain the tumorigenesis and development of SKCM and reduce cancer mortality, we further studied the molecular mechanism of SKCM.

The article "miR-100-5p Is a Novel Biomarker That Suppresses the Proliferation, Migration, and Invasion in Skin Cutaneous Melanoma" was retracted in 2023. Reasons: signs of a paper mill; suspected computer-generated content; unreliable results or conclusions; lack of ethics approval or compliance.

MicroRNAs (miRNAs), which regulated gene expression as posttranscriptional negative regulators of mRNAs encoding proteins, are thus well known and are small noncoding RNAs comprising 19-25 nucleotides. It is estimated that more than half of human mRNAs is a conserved miRNA target. Also, miRNAs are critical in many cellular processes in tumor cells, from differentiation and proliferation to death, and are tumor suppressor genes or oncogenes [3]. Numerous studies in SKCM have shown that miRNAs are aberrantly expressed, modulating proliferation, invasion, and metastasis of tumor cells [4, 5]. Meanwhile, miRNAs not only are regulators for neoplasm biological characteristics but also influence tumor microenvironment (TME) and enhance immunotherapy response [6]. For example, miR-21 can reduce the activity of T cells and promote cancer associate fibroblasts by targeting STAT1 and SMAD7 and reduce the response to antiprogrammed death in SKCM [7, 8].

MicroRNA-100-5p (miR-100-5p) is a highly conserved miRNA located on chromosome 11q24.1. Based on previous studies, several cancer cells have aberrant miR-100-5p presentation. It has been suggested to play multiple and, in some cases, contradictory roles in cancers, including breast cancers, prostate cancers, stomach adenocarcinoma, and chordoma [9–12]. However, how miR-100-5p in SKCM exerts a function is unclear, which still requires further exploration. In this research, the relation and clinical features between miR-100-5p expression were explored by us, and this study measured how miR-100-5p worked on tumor immune infiltration. We assessed the significance of miR-100-5p and then confirmed it with in vitro experiments. According to risk factors, furthermore, we constructed prognostic patterns and miR-100-5p expression to predict the disease-free interval and overall survival. Finally, a ceRNA network was constructed to reveal the miR-100-5p upstream-downstream regulatory mechanisms. We evaluated the underlying function of miR-100-5p and then revealed that it served as a prognostic and immune-related biomarker in SKCM, which may be considered an attractive molecular target for SKCM therapy in the future.

## 2. Materials and Methods

### 2.1. Data Collection and Clinical Correlation Analysis of miR-100-5p

We collected miRNA and gene expression profile information of patients from The Cancer Genome Atlas (TCGA) database. We analyzed a sample of 450. We gained clinical information on SKCM patients from the metadata option.  Table 1 shows the baseline clinical characteristics of patients in TCGA-SKCM. We downloaded chip per kilobase data (FPKM), and we modified them to transcripts per kilobase million (TPM) and log2 (TPM + 1). R packages “ggplot2” were used for visualization of relevance between clinical data and miR-100-5p, involving melanoma ulceration, TNM phrase, melanoma Clark level, and Breslow depth. We used the R packages “survival” and “survminer” to visualize and analyze miR-100-5p.

The article "miR-100-5p Is a Novel Biomarker That Suppresses the Proliferation, Migration, and Invasion in Skin Cutaneous Melanoma" was retracted in 2023. Reasons: signs of a paper mill; suspected computer-generated content; unreliable results or conclusions; lack of ethics approval or compliance.

### 2.2. Cell Lines and Cell Culture

From the American Type Culture Collection (ATCC), we took A375 and A2508 (SKCM cell lines). Using high glucose Dulbecco's modified Eagle medium (DMEM) (Gibco, Grand Island, NY, USA), this study separately cultivated the cells. We supplied all fresh media with 10% fetal bovine serum (Gibco) and antibiotics (Gibco). We routinely cultured A375 and A2508 cells in an incubator humidified with 5% CO_2_ at 37°C. The conventional cell culture methods are primary culture and subculture. We selected cells with a good culture environment for later study.

### 2.3. Cell Transfection and Real-Time Quantitative Polymerase Chain Reaction (qRT-PCR)

GenePharma Ltd. (Shanghai, China) synthesized the negative control for miR-100-5p inhibitor (inhibitor-N.C.) and miR-100-5p inhibitor (inhibitor), miR-100-5p negative control (control), miR-100-5p overexpression and inhibition in A375 and A2508 cell lines, miR-100-5p-mimic (mimic), and negative control for miR-100-5p mimics (mimic-N.C.). Using Lipofectamine 2000 (Invitrogen, New York, USA), this experiment was based on the manufacturer's instructions and transfected the sequences into cells. After transfection, this experiment carried out qRT-PCR to recognise the transfection influence. With Steponeplus Real-Time PCR System and the SYBR-Green PCR Master Mix kit, qRT-PCR was studied, and U6 expression was applied to be a domestic reference control for miR-100-5p. We used the 2-*ΔΔ*Ct approach to measure the gene expression's relative quantification. Three biological replicates made up each experiment. For each biological sample, we performed three technical replicates. For each gene, the primers are presented: miR-100-5p: F: 5′-GAACCCGTAGATCCGAACT-3′, R: 5′-CAGTGCGTGTCGTGGAGT-3′; U6: F: 5′-CTCGCTTCGGCAGCACA-3′, R: 5′-AACGCTTCACGAATTTGCGT-3′.

### 2.4. Cell Proliferation Assay

In 96-well plates, we conducted proliferation capacity by using the Cell Counting Kit-8 (CCK-8) (Biotechwell, Shanghai, China). Briefly, this study seeded 2∗10^3^ cells in 96-well plates cultivated for 24, 48, 72, and 96 hours. Then, 10 *μ*L CCK-8 solution after that was added to each well and incubated, lasting two hours at 37°C. With a microplate reader, we calculated the optical density (OD) at 450 nm (Thermo Fisher Scientific, Waltham, MA, USA). Experiments were performed in a minimum of three replicates.

The article "miR-100-5p Is a Novel Biomarker That Suppresses the Proliferation, Migration, and Invasion in Skin Cutaneous Melanoma" was retracted in 2023. Reasons: signs of a paper mill; suspected computer-generated content; unreliable results or conclusions; lack of ethics approval or compliance.

### 2.5. Flow Cytometry for Apoptosis Analysis

Through flow cytometry and Annexin V-PI staining, this study evaluated apoptosis. Briefly, according to the manufacturer's instructions, we used the Annexin V/FITC Kit (BD Biosciences, CA, USA) for staining of A2508 and A375 cells. Annexin V+/PI+ cells were regarded as late apoptotic cells, while Annexin-V (+)/PI(-) cells were regarded as apoptotic cells at the early stage. We evaluated the fraction of early apoptotic and late apoptotic cells through flow cytometry (BD Biosciences, San Jose, CA, USA).

### 2.6. Transwell Assay

In a 24-hole, 8 *μ*m interwell transwell, the invasion ability of the cells was determined by the transwell assay. After transfection, 2 × 10^4^ A375 and A2508 cells and their negative control cells were cultured in the upper chamber in 200 *μ*L serum-free medium. Meanwhile, add 700 *μ*L of fresh absolute medium to the lower chamber. After 24 hours of incubation, 1 mL of 4% formaldehyde solution was added to each well and allowed to stand for 15 minutes at room temperature. We used 0.5% crystal violet to stain migrating cells (Sinopharmatic Chemicals, China) and their photo microscope (Olympus). ImageJ software was used to calculate and limit the number of migrating cells. All experiments were repeated at least three times.

### 2.7. Scratch Wound Healing Assay

By the wound healing (scratch) assay in 6-well plates, we identified the cell migration capacity. Briefly, 1 × 10^6^ cells were seeded, and through a 1000 *μ*L sterile plastic pipette tip, a 1 cm width scratch segment was developed. The scratches were imaged at each time point (24 h, 48 h) to measure the cellular movement into the scratch. The percentage of the reduced scratch area to the original scratch area is the cell migration capacity. This study applied ImageJ software to measure the wound area, and all experiments were performed three times.

### 2.8. Analysis of the Relationship between Tumor Microenvironment and miR-100-5p

According to miR-100-5p expression, we split SKCM samples into 2 groups in order to explore its effect on the tumor microenvironment (TME). Based on their gene signatures, we used the ssGSEA algorithm of the built-in R package “GSVA” (version 1.34.0) to study its abundance [13]. We utilized the R package “Estimation” (version 1.0.13) to measure the composite score, containing the immunization value, substrate value, and estimation value. At the same time, the correlation between each TME cell and the miR-100-5p was calculated and visualized using R software.

The article "miR-100-5p Is a Novel Biomarker That Suppresses the Proliferation, Migration, and Invasion in Skin Cutaneous Melanoma" was retracted in 2023. Reasons: signs of a paper mill; suspected computer-generated content; unreliable results or conclusions; lack of ethics approval or compliance.

### 2.9. Construction and Evaluation of Prognostic Model

We predicted the disease-free interval and overall survival probability of SKCM by means of a prognostic nomogram model. Clinical factors and miR-100-5p expression were included in the nomogram. miR-100-5p was calculated using the formula log2(reads per million mapped reads + 1). By multivariate Cox regression methods, we measured overall survival at 1, 3, and 5 years. We used calibration plots to measure nomogram model performance. Through “survival” (version 3.2-10) and R packages “rms” (version 6.2-0), calibration plots were constructed.

### 2.10. Construction of the Regulatory Network of miR-100-5p

Target mRNA of miR-100-5p was forecasted using TargetScan v8.0 [14], miRDB [15], and miRTarBase v9.0 [16]. The target lncRNA for miR-100-5p was predicted using miRcode v11 (http://www.mircode.org/). The genes which negatively correlated with miR-100-5p were considered meaningful targets. The String v11 database [17] was used to obtain an interaction network among target mRNAs (confidence score > 0.7). Utilizing the R package “clusterProfiler” (version 3.14.3), functional enrichment analysis was carried out by us. Also, we formed the lncRNA-miRNA-mRNA regulatory network through Cytoscape software (version 3.8.2).

### 2.11. Statistical Analysis

The miR-100-5p expression was calculated using log2 transformation of reads per million mapped reads (RPM). We analyzed statistics by using R software (version 3.6.3) and GraphPad Prism 9.0 and used the chi-squared test and Wilcoxon rank-sum test to measure the correlation between miR-100-5p presentation and clinical data. Student's *t*-test and one-way ANOVA were applied to compare the significance between experimental groups,

## 3. Results

### 3.1. miR-100-5p Downregulation Is Associated with a More Aggressive Clinical Behavior of SKCM

Given the multiple roles of miR-100-5p in cancer behavior, we intended to understand its biological function in SKCM. We used bioinformatics analysis and found that miR-100-5p expression was closely correlated with T phase, N phase, Breslow's deep ulcer, and Clark level. However, there was no statistically significant correlation with M phase (Figures 1(a)–1(f)).  Table 2 shows the multivariate Cox regression results of some risk factors, showing that miR-100-5p in SKCM can be considered an independent risk factor for overall survival. Meanwhile, Kaplan-Meier survival analysis showed that low miR-100-5p expression was associated with decreased overall survival (Figure 1(g)), disease-specific survival (Figure 1(h)), and progression-free interval (Figure 1(i)). According to all the results of miRNA sequencing analysis, there was a significant correlation between the low expression level of miR-100-5p and the invasive behavior of SKCM.

The article "miR-100-5p Is a Novel Biomarker That Suppresses the Proliferation, Migration, and Invasion in Skin Cutaneous Melanoma" was retracted in 2023. Reasons: signs of a paper mill; suspected computer-generated content; unreliable results or conclusions; lack of ethics approval or compliance.

### 3.2. miR-100-5p Dysregulation Affects SKCM Cell Proliferation, Apoptosis, Invasion, and Migration

We transfected A375 and A2508 with miR-100-5p mimics, miR-100-5p inhibitors, and negative controls. We determined the role of miR-100-5p in SKCM.  Figure 2(a) shows the overexpression and inhibition efficiency of miR-100-5p verified by qPCR. CCK-8 results showed that compared with the control group, the growth of SKCM cells in the simulation group was inhibited by overexpression of miR-100-5p (Figures 2(b) and 2(c)). Figures 2(d) and 2(e) suggest that miR-100-5p could significantly trigger cell apoptosis, and apoptosis was inhibited when miR-100-5p was inhibited. In terms of invasion ability, transwell found (Figures 3(a) and 3(b)) that miR-100-5p overexpression inhibited SKCM cell invasion, while the invasion ability of SKCM cells in the miR-100-5p inhibitor group was decreased. Wound healing experiments (Figures 3(c) and 3(d)) showed that downregulation of miR-100-5p significantly enhanced the migration ability of cells at 24 h and 48 h. They tended to upregulate miR-100-5p to inhibit cell metastasis, but not significantly. Together, these data suggest that miR-100-5p plays a synergistic role in the inhibition of SKCM progression.

### 3.3. The Effects of miR-100-5p on Tumor Microenvironment

We compared the abundance of immune-related cells with low and high miR-100-5p expression and further investigated the significance of miR-100-5p on TME. After the analysis of this experiment, immune cell infiltration was achieved, including T helper cells, Th1 cells, T central memory cells (Tcm), *γδ*T cells (Tgd), CD8+ T cells, B cells, NK cells, and macrophages, which were significantly increased when miR-100-5p was highly expressed (Figure 4(a)). Interestingly, when miR-100-5p expression was higher (log2(RPM + 1) > 12.5), there was a positive correlation between miR-100-5p and TME.  Figure 4(b) shows the correlation between representative immune cells and miR-100-5p expression. Similarly, the same trend was more pronounced in the matrix score, immune score, and estimation score (Figures 4(c) and 4(d)), indicating that the effect of miR-100-5p on TME was bidirectional.

### 3.4. The Individualized Prediction Model Based on the Risk Signature and miR-100-5p Expression

We construct a prediction model since the biological behavior of SKCM cells might be dysregulated by miR-100-5p based on age, TNM staging, and miR-100-5p expression level. After excluding the samples with missing clinical information, 314 samples were included in the prognostic analysis. The nomograms were constructed based on the clinical information of the above patients to predict both overall survival and disease-free survival probability (Figures 5(a) and 5(c)). The calibration curves run close to the ideal calibration line, which shows a satisfactory prediction accuracy for 1-, 3-, and 5-year overall survival rates (Figures 5(b) and 5(d)).

The article "miR-100-5p Is a Novel Biomarker That Suppresses the Proliferation, Migration, and Invasion in Skin Cutaneous Melanoma" was retracted in 2023. Reasons: signs of a paper mill; suspected computer-generated content; unreliable results or conclusions; lack of ethics approval or compliance.

### 3.5. The lncRNA-miRNA-mRNA Regulatory Network of miR-100-5p

We predicted the related lncRNAs and mRNAs of miR-100-5p through the public database to understand its upstream and downstream regulatory relationship. Through R software, we found that the expressions of 2707 mRNAs and 129 lncRNAs were negatively correlated with miR-100-5p. After taking the intersection of negatively correlated mRNAs and target genes predicted by TargetScan, miRDB, and mirTarbase, we identified 58 downstream candidate mRNAs (Figure 6(a)). GO/KEGG analysis showed that these 58 mRNAs were mainly enriched in mitochondria, respiratory chain, and G2/M phase transition function of the cell cycle (Figure 6(b)). Next, we took the intersection of negatively correlated lncRNAs predicted by the miRcode database and target genes. Four upstream lncRNAs were identified as candidate lncRNAs (Figure 6(c)), including AP002748.4, LINC01315, AC027237.3, and AC008915.3. The ceRNA regulatory network and PPI network between target mRNAs are shown in Figure 6(d).

## 4. Discussion

Malignant melanoma represents one of the most life-threatening skin cancers worldwide and one of the most likely malignancies to metastasize [18]. However, the molecular mechanism of its malignant behavior is not yet known. Recently, miRNA was regarded to act as a significant role in tumor progression, including SKCM [4, 5, 19]. miR-100-5p has been proved to have an impact on the biological behavior of some tumors. For example, chordoma has a low miR-100-5p expression, and also targeting IGF1R restrains the malignant activity [20]. In stomach adenocarcinoma, miR-100-5p is an independent risk factor and a prognostic marker to predict the survival time [11]. In SKCM, however, miR-100-5p function and its modulatory working principles were not fully validated in SKCM. This experiment discovered that miR-100-5p was significantly correlated with malignant behaviors of SKCM, which is also associated with SKCM patients' disease-specific survival and overall survival and progress-free interval. However, the relationship between M stage and miR-100-5p presentation was not statistically significant, suggesting basically that the miR-100-5p was engaged in local invasion rather than distant metastasis in SKCM. In A375 and A2508 cells, additionally, we performed both miR-100-5p inhibition and overexpression assay. In this experiment, notably, as miR-100-5p was overexpressed, cell propagation, aggression, and moving were restrained, but apoptosis was improved. And when miR-100-5p was restrained, cell propagation, aggression, and moving were accelerated, but apoptosis was restrained.

miRNAs can not only influence tumor progression but also regulate the landscapes of TME [6]. Szczepaniak Sloane et al. discovered that miR-100-5p was related to PD-1 checkpoint blockade outcomes and may serve as a potential immunotherapy target [21]. Therefore, this study explores miR-100-5p significance in the immune infiltration of SKCM. Generally, the abundance of cytotoxic T lymphocytes (CD8+ T cells), tertiary lymphoid structures, and B cells indicates a good prognosis. In contrast, the abundance of regulatory T cells (T-reg cells) and macrophages (especially M2 macrophages) indicates a bad prognosis in melanoma [22]. This experiment suggested that miR-100-5p can elicit infiltration of immunity in the local environment using ssGSEA and ESTIMATE algorithm. However, it is noteworthy that upon further analysis of the relation between miR-100-5p expression and TME scores, the impact of miR-100-5p on TME appeared to be bidirectional. The tumors with the intermediate miR-100-5p expression have the highest immune cell infiltration levels, indicating that these patients may have a preferential reaction to immunotherapy. However, because of tumor immunity complexity, the specific mechanism of the miR-100-5p influence on TME needs further exploration.

The article "miR-100-5p Is a Novel Biomarker That Suppresses the Proliferation, Migration, and Invasion in Skin Cutaneous Melanoma" was retracted in 2023. Reasons: signs of a paper mill; suspected computer-generated content; unreliable results or conclusions; lack of ethics approval or compliance.

Whether the tumor has progressed or not seems to be one of the biggest concerns for patients. Therefore, we hope to construct a prognostic model to predict tumor progression in SKCM. Because the abnormal regulation of miR-100-5p can greatly affect the malignant behavior of tumors, a model was constructed according to the clinical characteristics and the expression level of miR-100-5p. By adding each patient's risk factors, overall disease-free interval, and SKCM scores at 1, 3, and 5 years, we could predict their probability of survival. The calibration curves prove that the two models have good prediction accuracy. Using this prognostic model, the physician can adjust the follow-up time according to the clinical characteristics of the patient.

The ceRNA network was constructed to reveal the regulatory miR-100-5p relationships. Since lncRNAs and miRNA are able to serve as molecular sponges of downstream genes [23], the predicted genes that negatively correlated with miR-100-5p expression were identified as target genes. Functional enrichment analysis shows that the downstream mRNA is mainly associated with mitochondria metabolism and cell cycle transition. The dysregulation of mitochondrial function is essential for the occurrence of cancer cell proliferation and invasion. Meanwhile, the ATP production of the G2/M phase mainly depends on mitochondrial respiration. Inhibition of the mitochondrial function in the G2/M stage leads to cycle stagnation [24]. In melanoma, there was a correlation between high expression of mitochondrial biogenesis and poor prognosis [25, 26]. The insufficient expression of miR-100-5p may cause mitochondrial dysfunction, leading to further activation of G2/M phase transition and cell proliferation. We also identified four lncRNAs that have regulatory relationships with miR-100-5p. Among them, LINC01315 proved to act as a molecular decoy of miRNAs and promote malignant cell behaviors in diverse cancers, like colorectal cancer [27], breast cancer [28], and thyroid cancer [29]. Nevertheless, functions of AP002748.4, AC027237.3, and AC008915.3 in cancers remain to be clarified.

The article "miR-100-5p Is a Novel Biomarker That Suppresses the Proliferation, Migration, and Invasion in Skin Cutaneous Melanoma" was retracted in 2023. Reasons: signs of a paper mill; suspected computer-generated content; unreliable results or conclusions; lack of ethics approval or compliance.

We improve the understanding of the relationship between miR-100-5p and SKCM. However, several limitations need to be addressed. First, although we constructed a regulatory network and explored the correlation between miR-100-5p and tumor microenvironment, these linkages lack direct experimental confirmation. Furthermore, we did not perform directly in vivo experiments to extrapolate our findings to the in vivo environment.

In summary, we were able to predict the probability of survival for each patient by adding their risk factors, overall disease-free interval, and SKCM scores at 1, 3, and 5 years compared to previous studies. This further elucidated that tumors with intermediate miR-100-5p expression had the highest level of immune cell infiltration, suggesting that these patients may have a preferential response to immunotherapy. However, due to the complexity of tumor immunity, the specific mechanism of miR-100-5p affecting TME needs to be further explored.

## 5. Conclusion

In general, antitumor miR-100-5p effect and its molecular regulatory network were revealed in this study. The immune microenvironment analysis and the prediction nomogram model confirmed the translational use of miR-100-5p in SKCM immunotherapy and immunotherapy.

## Figures and Tables

**Figure 1:** Lower miR-100-5p expression was associated with higher tumor stage and lower survival rates: (a–f) the correlation between miR-100-5p expression and clinical parameters, including (a–c) TNM stage, (d) Breslow depth, (e) melanoma ulceration, and (f) melanoma Clark level; (g–i) Kaplan-Meier survival analyses of miR-100-5p in SKCM patients on (g) overall survival, (h) disease-specific survival, and (i) progress-free interval (^∗^*p* < 0.05,  ^∗∗^*p* < 0.01, and^∗∗∗^*p* < 0.001).

The article "miR-100-5p Is a Novel Biomarker That Suppresses the Proliferation, Migration, and Invasion in Skin Cutaneous Melanoma" was retracted in 2023. Reasons: signs of a paper mill; suspected computer-generated content; unreliable results or conclusions; lack of ethics approval or compliance.

**Figure 2:** miR-100-5p dysregulation affects SKCM cell proliferation and apoptosis. (a, b) Transfection efficiency of (a) miR-100-5p-mimic and (b) miR-100-5p-inhibitor was confirmed using qRT-PCR in A2508 and A375 cell lines. (c, d) Cell proliferation ability was evaluated by CCK-8 assay in (c) A2508 and (d) A375 cell lines. (e, f) Cell apoptosis was evaluated by flow cytometry analysis in (e) A2508 and (f) A375 cell lines (^∗^*p* < 0.05,  ^∗∗^*p* < 0.01, and^∗∗∗^*p* < 0.001).

**Figure 3:** miR-100-5p dysregulation affects SKCM cell invasion and migration. (a, b) Cell invasion ability was evaluated by transwell assay in (a) A2508 and (b) A375 cell lines. (c, d) Cell migration ability was evaluated by scratch wound healing assay in (c) A2508 and (d) A375 cell lines (^∗^*p* < 0.05,  ^∗∗^*p* < 0.01, and^∗∗∗^*p* < 0.001).

**Figure 4:** The influence of miR-100-5p on the tumor microenvironment. (a) The abundance of immune-related cells in miR-100-5p high- and low-expressed groups was evaluated by the ssGSEA algorithm. (b) The correlation between miR-100-5p expression and immune cells. (c) The tumor microenvironment scores in miR-100-5p high- and low-expressed groups were evaluated by the ESTIMATE algorithm. (d) The correlation between miR-100-5p and the tumor microenvironment scores (^∗^*p* < 0.05,  ^∗∗^*p* < 0.01, and^∗∗∗^*p* < 0.001).

**Figure 5:** Construction and assessment of prognostic nomogram of disease-free interval and overall survival. (a, c) The nomogram for predicting 1-, 3-, and 5-year disease-free interval and overall survival. The survival probability was predicted using total points calculated by adding up the score of each risk factor. (b, d) The calibration plots for validating 1-, 3-, and 5-year disease-free interval prediction. The diagonal is the ideal calibration line. The curve in good agreement with the ideal line accurately predicts survival probability.

**Figure 6:** The regulatory network of miR-100-5p in SKCM: (a) the Venn diagram shows that 58 mRNAs were the downstream targets of miR-100-5p in SKCM; (b) the functional enrichment analysis of 58 selected mRNAs; (c) the Venn diagram shows that 4 lncRNAs were the upstream targets of miR-100-5p in SKCM; (d) the regulatory network of miR-100-5p.

**Table 1:** The baseline clinical characteristics of TCGA-SKCM.

Characteristic	Levels	Low expression of hsa-miR-100-5p	High expression of hsa-miR-100-5p	*p*
Gender, *n* (%)	Female	84 (18.7%)	88 (19.6%)	0.771
	Male	141 (31.3%)	137 (30.4%)	

Age, *n* (%)	≤60	109 (24.7%)	135 (30.5%)	0.013
	>60	113 (25.6%)	85 (19.2%)	

T stage, *n* (%)	T1	21 (6.1%)	17 (4.9%)	<0.001
	T2	31 (9%)	48 (13.9%)	
	T3	35 (10.1%)	50 (14.5%)	
	T4	93 (27%)	50 (14.5%)	

N stage, *n* (%)	N0	113 (28.3%)	113 (28.3%)	0.005
	N1	27 (6.8%)	43 (10.8%)	
	N2	20 (5%)	29 (7.3%)	
	N3	37 (9.3%)	17 (4.3%)	

M stage, *n* (%)	M0	197 (46.5%)	203 (47.9%)	0.513
	M1	14 (3.3%)	10 (2.4%)	

Breslow depth, *n* (%)	≤3	74 (21.6%)	106 (31%)	<0.001
	>3	100 (29.2%)	62 (18.1%)	

Melanoma ulceration, *n* (%)	No	66 (22.1%)	75 (25.1%)	0.008
	Yes	99 (33.1%)	59 (19.7%)	

Melanoma Clark level, *n* (%)	I	2 (0.7%)	4 (1.3%)	0.003
	II	9 (2.9%)	8 (2.6%)	

The article "miR-100-5p Is a Novel Biomarker That Suppresses the Proliferation, Migration, and Invasion in Skin Cutaneous Melanoma" was retracted in 2023. Reasons: signs of a paper mill; suspected computer-generated content; unreliable results or conclusions; lack of ethics approval or compliance.

**Table 2:** The univariate Cox regression of risk factors in SKCM.

Characteristics	Total (*N*)	Univariate analysis		Multivariate analysis	
		Hazard ratio (95% CI)	*p* value	Hazard ratio (95% CI)	*p* value
T stage	342				
T1	38	Reference			
T2	77	1.542 (0.807-2.946)	0.190	1.924 (0.941-3.935)	0.073
T3	84	2.240 (1.189-4.221)	0.013	2.927 (1.177-7.277)	0.021
T4	143	3.895 (2.085-7.279)	<0.001	5.571 (2.261-13.726)	<0.001
N stage	387				
N0	215	Reference			
N1	69	1.572 (1.057-2.339)	0.026	2.989 (1.019-8.772)	0.046
N2	49	1.529 (0.967-2.415)	0.069	3.026 (1.003-9.130)	0.049
N3	54	2.730 (1.754-4.250)	<0.001	6.675 (2.182-20.424)	<0.001
M stage	411				
M0	388	Reference			
M1	23	1.752 (0.923-3.323)	0.086	0.612 (0.149-2.509)	0.495
Pathologic stage	389				
Stage I	75	Reference			
Stage II	128	1.646 (1.079-2.511)	0.021	0.733 (0.350-1.538)	0.411
Stage III	164	2.129 (1.431-3.168)	<0.001	0.425 (0.128-1.411)	0.162
Stage IV	22	3.401 (1.672-6.916)	<0.001		
hsa-miR-100-5p	435	0.859 (0.795-0.927)	<0.001	0.873 (0.797-0.958)	0.004

## Data Availability

The experimental data used to support the findings of this study are available from the corresponding authors upon request.
